# Biomechanical Analysis of Touch Ball Movements in Tennis Forehand Strokes

**DOI:** 10.1155/2022/5754820

**Published:** 2022-06-16

**Authors:** Wufeng Luo

**Affiliations:** Department of Physical Education, Guangdong Pharmaceutical University, Guangzhou, Guangdong 510006, China

## Abstract

In order to improve the effect of certain theoretical basis for tennis coaches to correct technical movements and teaching training, a method oriented towards discrete gradient methods that can be used for computational solid mechanics is presented. The biggest feature of this method is that it can directly perform numerical simulation analysis on any point cloud model, without relying on any structured or unstructured grid model. Experimental results show that about 80% of the shots in the game are within 2.5 m of the athlete's moving distance, and the athlete needs to have 300 to 500 high-intensity exercises; the total running distance of the competition is 1 100–3 600 m. The average VO2 of athletes during the competition is 20–30 mL/min/kg (45%–55% V.O2max), the average heart rate is 135–155 beats/min (70%–85% HRmax), the mean blood lactate was <4 mmol/L, the subjective fatigue was 12–14 (moderate intensity), and the mean metabolic equivalent was 5–7 METs. It is proved that the discrete gradient method can effectively solve the biomechanical analysis problem of tennis forehand hitting the ball. Make up for the lack of action details in the differentiation stage. Improve the effect of certain theoretical basis for tennis coaches to correct technical movements and teaching training.

## 1. Introduction

Tennis is a highly technical sport; it not only is a sport for large muscle groups, but also involves many small muscle groups; therefore, it is very easy to make various mistakes in the process of improving the level of tennis skills. If these wrong actions cannot be corrected in time, it will affect the learner's mastery of the complete technique and even lead to injury. Therefore, to correct wrong actions scientifically and effectively, as an important problem to be solved in tennis learning, biomechanics is the study of human movement. In terms of physical mechanics, the perfect technique of tennis is the effective combination of maximum force and control and minimizes the chance of injury. A biomechanic studies tennis technique, by determining the most effective types of moves necessary to form a play, analyze the effectiveness of a practitioner's movements, and try to determine if he can perform them more effectively. When analyzing and correcting movements, a proper understanding of cow physics will help coaches avoid focusing on the performance of the hitting action; instead, it focuses more on the effectiveness of the shot [1].

The basic technical movements of tennis include serving, forehand and backhand, and volley; in the modern tennis sport where the bottom line is the mainstream, forehand is the most important technical action after serving in various tennis techniques; studies have shown that, in the game, forehand hits are about 25% more often than backhand hits. Forehand is divided into closed forehand and open forehand; closed forehand requires players to have their feet perpendicular to the bottom line when hitting the ball; in the process of hitting the ball, the center of gravity of the body can be transferred from the back to the front, so that the power and speed of the shot can be greater; in a long period of time, the closed style of hitting the ball was once considered the best way to hit the ball [2]. However, with the improvement of tennis forehand technical movements and the change of racket materials, more and more tennis players are using open strokes as the main way to hit the ball, because the feet are almost parallel to the bottom line when hitting the ball with the open footwork; the upper step is omitted compared with the closed footwork, allowing players to save batting time and be able to return quickly after hitting the ball. Moreover, in the forehand and backhand confrontation on the bottom line, the open footwork can play a strong topspin, reduce the hitting of the net and out of bounds, and at the same time increase the difficulty of the opponent's return, posing a greater threat to the opponent.

Tennis is a skill-oriented confrontational project with net separation, and the level of technical movements directly determines the performance of tennis players themselves. For the tennis public, tennis technical movements are more complicated than other sports, and it is not easy to master them quickly. Forehand is the first step in learning tennis, and learning the forehand can help improve confidence and experience the fun of tennis. And tennis is a whole-body sport, the power of hitting the ball comes from the lower limbs, and the arm swings through the rotation of the hips and shoulders; when hitting the ball, the upper and lower limbs need to coordinate and cooperate, and any link may affect the quality of the shot. According to the theory of sports training, the learning of technical actions needs to go through four stages: generalization, differentiation, consolidation and improvement, and automation; however, most tennis players in the ordinary group need to correct the details of their movements in the differentiation stage; if it is not corrected or the problems of its own movements cannot be found, the wrong movements will be brought to the next stage in repeated exercises, which will make it difficult to improve the technical level and even cause musculoskeletal joint damage [3].

At present, motion capture and analysis technology has been widely used in various sports, from football to swimming, from tennis to golf, from track and field to basketball, covering almost all sports. Through the measurement and evaluation of athletes' technical movements, it can help them improve their technical level and correct and optimize special movements, so as to prevent injuries and improve sports performance. At present, most of the literature focus on the research on the kinematic characteristics of the upper limbs of tennis forehand movements; there is still insufficient research on the whole-body kinematics and dynamic characteristics of the forehand movements of tennis players; it is impossible to provide comprehensive theoretical guidance to coaches and athletes and mainly rely on experience to teach and train forehand technical movements [4]. Therefore, the author analyzes the biomechanics of the tennis forehand and touch action by establishing a whole-body biomechanical model and provides a certain theoretical basis for tennis coaches to correct technical movements and teach training.

## 2. Literature Review

A forehand is usually divided into three phases, four key moments of action. First of all, in the back-swing lead-in phase, the shoulders are turned away from the net from the start to the end of the backward movement of the racket; at this stage, the racket moves backwards and the muscles of the upper limbs are stretched and elongated. The second stage is the forward acceleration swing stage, which starts when the racket moves forward for the first time and lasts until the moment of contact with the ball. During the forward swing of the racket, the upper and lower limbs form a dynamic chain, and the ground rotation drives the racket to continuously increase the speed of the racket head. The third stage is the postswing phase from the moment of contact to the end of the forward swing, during which the upper limb-racket complex is decelerated.

The difficulty of the forehand action is how to coordinate the lower limbs and upper limbs, because the lower limbs mainly push and stretch in the sagittal plane, while the trunk and upper limbs rotate in the horizontal plane. When hitting a forehand, you need to pay attention to the angle between the racket and the ground at the moment of hitting, which may affect the control of the flight path of the ball. When hitting the ball, the rotation of the body is accompanied by the movement of the center of gravity of the body; it is also necessary to choose the type of shot. For different shot types, control the angle between the racket and the ground; the angle between the racket and the ball is at the moment of contact; it produces the effect of topspin or flat strike [5]. See Figure 1.

Tennis players' forehand stance is usually divided into open stance and closed stance: In the open stance, the player's feet and hips are parallel to and facing the net, while in the closed stance, the player rotates almost 180°, and feet and hips are perpendicular to the net. There is currently no empirical data to quantify how professional tennis players play; using the ratio of different stances, Rusdiana proposed that 90% of forehand shots of high-level tennis players use open stance [6]. However, there are also studies pointing out that the relative distribution of forehand stance may be affected by gender, age, skill level, and court surface (hard/grass/clay). The open style of hitting the ball is flexible, it is easy to observe the opponent's situation when hitting the ball, and the return position is quick after hitting the ball. Closed batting footwork means that the feet are parallel to the hitting direction when hitting the ball, which can make the athlete's center of gravity move towards the hitting direction. During a closed shot, the athlete's center of gravity shifts to the direction of the shot to increase the power and speed of the shot. Chen argues that, with open footwork, before the athlete hits the ball, its body has made a large rotation from the legs to the shoulders and accumulated a lot of energy, which is also beneficial to the improvement of the hitting speed [7]. This angle of rotation is twice that of closed footwork, and the muscle groups of the waist and thighs are also fully engaged. Open footwork can easily apply topspin to the ball during hitting, and its running range is much smaller than that of closed footwork, open footwork requires athletes to have a higher technical level, because the hitting action requires very little time, and although the closed footwork is powerful and powerful, it is not easy to hit the ball with topspin.

Whether open stance and closed stance will affect the hitting speed and joint force, Fillmore and Hall think that open stance will cause a greater load on the athlete's body; however, some studies have also found that closed stance forehands have greater peak shoulder internal rotation torque and greater peak wrist flexion torque; this is in contrast to the idea that open stance shots place a greater load on the upper body [8]. Fleming et al. study the characteristics of trunk muscle activation during open and closed forehand strokes in tennis; the results of the study do not support the hypothesis that open poses produce greater trunk muscle activation than closed poses; the external oblique is important in axial rotation, and female tennis players may require greater external oblique activation due to fewer external oblique muscle fibers [9]. While Bankosz and Winiarski suggested that the upper extremity dynamics of the open and closed forehand are very similar, except for the peak torque in shoulder internal rotation and wrist flexion, all subjects developed shoulder internal rotation torque during the forward swing, and the closed shoulder internal rotation torque was significantly greater than the open one, and the wrist flexion torque was also significantly greater [10]. The data do not support the hypothesis that open forehands create significantly higher upper-body loads than closed ones. Instead, the closed forehand caused the subject to generate more torque, which resulted in a greater load at the joints. In addition, studies have also found that open and closed forehand footwork produce similar racket speed; in open forehand, because the center of gravity moves less in the direction of hitting, the speed of the center of the shoulder joint in the direction of hitting is lower than that in closed style; the force generated by the shoulder joint does less work in the direction of impact than with closed footwork. In open footwork, however, the torso rotates more in the direction of impact and has more upward acceleration; this results in the work done by the shoulder joint forces in the lateral and upward directions, more than you do in closed footwork, which makes up for the lack of shoulder work in the direction of impact in open footwork. In both poses, it was mainly the shoulder horizontal flexion moment and the shoulder internal rotation moment that increased the energy of the racket arm.

Tennis forehand grips include Eastern, Continental, Semi-Western, and Western grips; forehand skills are generally learned from the Eastern grip. With the improvement of tennis skills, the grip will also change accordingly. Some studies believe that the Western grip can not only produce greater speed than the Eastern grip, but also control the angle of the elbow joint. However, Zhang et al. proposed that the Western style grip will increase the probability of tennis elbow, because the pressure of the elbow valgus increases when the racket is accelerated. The Semi-Western grip, on the other hand, can not only handle the ball with low bounce, but also hit the ball with strong topspin, and the pressure on the elbow is relatively small when hitting the ball. The Semi-Western grip is between the Eastern and Western grips; this grip method enables athletes to handle most of the balls well; it can hit a strong topspin and handle low balls well, so it is loved by many players and has become the mainstream grip used by modern tennis players.

Each grip affects the kinematics of the athlete's forehand swing and therefore how the ball moves (topspin/flat/sidespin). Arul et al. found that forehand grip affects wrist injury in nonprofessional tennis players; over a 20-month monitoring period, approximately 13% of 370 tennis players reported grip-related wrist injuries, ulnar or radial wrist injuries, and pain associated with Eastern/Semi-Western/Western grips, respectively [11]. This is consistent with the study by Wahyudin et al.; Western and Semi-Western grips increase flexion of the ulnar wrist and also increase the vertical velocity of the racket. Therefore, when analyzing the causes of wrist injuries and proposing treatment methods for wrist injuries, the way of holding the racket must be considered [12].

When it comes to grip strength, tennis coaches often encourage players not to grip the racket too tightly, arguing that too much grip can lead to muscle tension, which can lead to slower swing speeds. But research has shown that grip strength has little effect on the speed of a simulated forehand return. In the process of swinging the racket to hitting the ball, the athlete can reduce the strength of the grip as long as the racket can be stabilized. However, Oshita et al. research shows that the grip strength of different parts of the palm varies greatly throughout the forehand stroke; grip strength increases in the 50 ms before the ball hits the face [13]. In addition, Maulidin et al. believed that increasing the grip strength may be unfavorable for hitting the ball in the central area of the racket head, and a strong grip of the forehand may reduce the flight time and trajectory of the ball after impact [14]. Obviously, these are all speculations, and further research is needed to fully understand the interaction between grip strength and forehand performance; there are also different grip techniques to take into account.

## 3. Method

### 3.1. Discrete Gradient Method

A discrete gradient method can be used for computational solid mechanics. The biggest feature of this method is that it is possible to perform numerical simulation analysis directly on any point cloud model, without relying on any structured or unstructured grid model. Discrete gradient method is done first through the relative displacement between adjacent points, in order to approximate the deformation gradient at each point; then, the system discretization equation is derived from the weak form through the deformation gradient, and the displacement, strain, and stress of each point in the model are finally calculated. Because there is no need to construct the continuous solution assumed in the finite element method or the meshless method, the operation process of the discrete gradient method is simple, the method is flexible, and the calculation efficiency is high. More importantly, the discrete gradient method can automate the process of image-based numerical simulation and software [15]. The author uses the discrete gradient method to derive the forehand based on tennis, biomechanical analysis of ball contact, in order to provide a convenient and practical tool for tennis coaches to correct technical movements and teaching training.

The discrete gradient method uses a generalized finite difference method to calculate the gradient of a function at discrete points. Compared with the classical finite difference method based on regular grid, the discrete gradient method can approximate the differential in a differential manner on an irregular grid or any discrete point cloud [16]. The specific derivation process of the discrete gradient method and the accuracy, stability, and convergence of the method have been described in detail in the literature.

In a point cloud model, if the volume represented by each point can be determined by the above method, then under the Lebesgue measure, the material volume thus defined can satisfy

(1) $$\begin{array}{c} \sum_{I}V_{I}=V, \end{array}$$

where *V* is the total volume of the point cloud model and *V*_*I*_ is the volume represented by point *I*. In order to distinguish the nodes in the finite element method, the points in the point cloud model are collectively referred to as material points in the following [17]. By dividing the center of gravity, the determined material point volume has an important characteristic; that is, in the rigid body motion, the translation invariance and the affine invariance under uniform deformation can be maintained, that is,

(2) $$\begin{array}{c} \left.\begin{array}{c} V_{I}\left(x_{I}+a,x_{J_{1}}+a,\ldots ,x_{J_{N}}+a\right)=\\ V_{I}\left(x_{I},x_{J_{1}},\ldots ,x_{J_{N}}\right),\forall a\in R^{3}\\ V_{I}\left(Fx_{I},Fx_{J_{1}},\ldots ,Fx_{J_{N}}\right)=\\ \det\left(F\right)V_{I}\left(x_{I},x_{J_{1}},\ldots ,x_{J_{N}}\right),\\ \forall \text{Linearmapping}F:R^{3}⟶R^{3},\det\left(F\right)\neq 0 \end{array}\right\}. \end{array}$$

If a material point *I* has *N*_*I*_ adjacent points, then the gradient interpolation vector at this point can be defined as follows:

(3) $$\begin{array}{c} R_{IJ}^{*}=\frac{1}{V_{1}}\frac{\partial V_{I}}{\partial x_{J}},J\in N_{I}. \end{array}$$

Then it can be proved that the defined gradient interpolation vector can satisfy the linear compatibility condition:

(4) $$\begin{array}{c} \sum_{J\in N_{I}}R_{IJ}^{*}=0,\\ \sum_{J\in N_{I}}R_{IJ}^{*}⊗x_{J}=I, \end{array}$$

where *I* is the same tensor of second order, and ⊗ represents tensor multiplication. The gradient interpolation vector definition method is not unique, and the adjacent relationship and volume of points determined by different geometric divisions are often different, but it does not affect the calculation process and accuracy [18].

Through the above definition, the gradient of the function *u* at point I can be discretized or approximated by the gradient interpolation vector as

(5) $$\begin{array}{c} {\left(\nabla^{h}u\right)}_{I}=\sum_{J\in N_{I}}R_{IJ}^{*}u_{J}. \end{array}$$

### 3.2. Application of Discrete Gradient Method in Biomechanical Analysis

If the position of the material point in the current configuration is *x*, and the position in the reference configuration is *x*, deformation Φ: *x* = Φ (*X*) can define the displacement of each point, so the deformation gradient of the material point I can be discretized as

(6) $$\begin{array}{c} F_{I}^{h}:={\left(\nabla^{h}\varphi \right)}_{I}\\ =\sum_{J\in N_{I}}x_{J}⊗R_{IJ}^{*}, \end{array}$$

where the interpolation vector *R*_*IJ*_^*∗*^ is defined in the reference configuration. The corresponding deformation gradient variation can be derived from the displacement variation

(7) $$\begin{array}{c} \delta F_{I}^{h}:={\left(\nabla^{h}\delta \varphi \right)}_{I}\\ =\sum_{J\in N_{I}}\delta \varphi_{J}⊗R_{IJ}^{*}. \end{array}$$

The discrete displacement variational spatial gradient can be expressed as

(8) $$\begin{array}{c} {\left(\nabla^{h}\delta \varphi \right)}_{I}=\left(\delta F_{I}^{h}\right){\left(\delta F_{I}^{h}\right)}^{-1}. \end{array}$$

By the Lagrangian method, the system equation of the boundary value problem is expressed as

(9) $$\begin{array}{c} \left.\begin{array}{c} DivP+\rho_{0}b=\rho_{0}\overset{¨}{u},PF=F^{T}P^{T},\text{in}\Omega_{0}\\ PF=\bar{p},on\partial \Omega_{ot}\\ \Phi =\bar{\Phi },on\partial \Omega_{ou} \end{array}\right\}, \end{array}$$

where *P* is the first Piola Kirchhoff stress, *b* is the body force per unit of matter, *u* is the displacement vector, *N* is the outer normal vector on the boundary, $\bar{p}$ is the applied load on the boundary, and the subscript 0 represents the reference configuration [19]. Then, the weak form of the boundary value problem can be derived as

(10) $$\begin{array}{c} \int_{\Omega_{0}}\nabla \delta \Phi :P\left(F\right)\text{d}V+\int_{\Omega_{0}}\delta \Phi \cdot \rho_{0}\overset{¨}{u}\text{d}V-\int_{\Omega_{0}}\delta \Phi \cdot \rho_{0}ub\text{d}A-\int_{\partial \Omega_{0t}}\delta \Phi \cdot \bar{\rho }\text{d}S=0, \end{array}$$

where ∂Φ is the virtual displacement. After discretization of the displacement gradient, the weak form can be approximated as

(11) $$\begin{array}{c} \sum_{I}V_{0I}{\left(\nabla^{h}\delta \Phi \right)}_{I}:P\left(F_{I}^{h}\right)+\sum_{I}V_{0I}\delta \Phi_{I}\cdot \rho_{0}{\overset{¨}{u}}_{I}\\ =\sum_{I}V_{0I}\delta \Phi_{I}\cdot \rho_{0}b_{I}+\sum_{I}A_{tI}\delta \Phi_{I}\cdot {\bar{p}}_{I}, \end{array}$$

where *A*_*tI*_ is the surface area of the element to which the external load is applied. For hyperelastic materials, the first Piola Kirchhoff stress can be obtained from the material's strain energy function W via *P*(*F*_*I*_)=*∂W*/*∂F*_*I*_. So it can be simplified to

(12) $$\begin{array}{c} \sum_{I}F_{I}^{\text{ext}}\cdot \delta \Phi_{I}. \end{array}$$

And

(13) $$\begin{array}{c} F_{I}^{\text{ext}}=V_{0I}\rho_{0}b_{I}+A_{tI}{\bar{p}}_{I}. \end{array}$$

In the formula, *F*_*I*_^ext^ corresponds to the external force acting on the material point *I*. The internal force *F*_*I*_^int^ of the node can be derived through the stress divergence term, so that

(14) $$\begin{array}{c} \sum_{I}\delta \Phi_{I}\cdot F_{I}^{\mathrm{int}}=\sum_{I}V_{0I}{\left(\nabla^{h}\delta \Phi \right)}_{I}:P\left(F_{I}^{h}\right). \end{array}$$

Combining the equations, the system of nonlinear equations derived in discrete weak form can be obtained

(15) $$\begin{array}{c} F_{I}^{\mathrm{int}}+m_{I}{\overset{¨}{u}}_{I}-F_{I}^{ext}=0. \end{array}$$

*m*_*I*_=*ρV*_0*I*_. The system of equations can be solved by the Newmark method in the time domain integration, and the calculation of the tangential stiffness matrix is consistent with the process in the finite element method [20].

The above calculation process is derived from the weak form; it has similar accuracy and convergence as the bilinear quadrilateral element in the finite element method and can pass the standard patch test.

### 3.3. Biomechanical Analysis of Wrong Actions When Touching the Ball

In the tennis forehand technique, when the racket is in contact with the ball, the four main links of the legs, hips, upper body, and head and shoulders coordinate with each other to construct the correct action when touching the ball and increase the power of returning the ball. The correct actions when touching the ball are shown in Table 1, and the wrong actions that are prone to occur are shown in Table 2.

## 4. Experimental Results and Discussion

### 4.1. Kinematic Characteristics of Arm Manipulation

Tennis is a highly professional sport, and high-level professional players need to participate in about 20 events and about 70 matches every year. The height of the world's top tennis players (men) is about 184 cm, the weight is about 79 kg, and the BMI is about 23.5 kg/m^2^; there is a certain gap between the height and weight of tennis players with low sports level. The V.O2max of tennis players is 46 to 72 mL/min/kg (male) and 42 to 52 mL/min/kg (female), which is lower than that of elite endurance athletes, but similar to those of other racket-holding athletes [21]. At low levels, athlete V.O2max appeared to be related to exercise level, but at high levels, V.O2max was not related to exercise level. The peak anaerobic power of adult tennis players is 10–12 W/kg (men) and 8–10 W/kg (women), which are weaker than those with higher exercise intensity. The tennis incremental run stroke test appears to be a simple and effective method for evaluating V.O2max in tennis players [22].

Tennis is an intermittent sport, and alternating between high-intensity hitting and intermittent rest is the basic feature of tennis. The duration of a tennis match is 1.5 to 5 hours, the average round time is 4 to 10 s, and the average interval between rounds is 10 to 25 s, the ratio of exercise to rest is 1 : 1 to 1 : 4, and the effective game time is 20% to 50%. In tennis, the average moving distance of each shot is 3 m, and the moving distance for each point is 8–15 m. It is necessary to complete 4 changes of direction, and the number of shots is 2–6 times [23]. About 80% of the shots in the game are within 2.5 m of the player's moving distance, and the player needs to do 300–500 high-intensity exercises, and the total running distance of the game is 1100–3600 m. See Figures 2 and 3.

The overall physiological intensity of tennis matches is not high. The average VO2 of athletes during the game is 20–30 mL/min/kg (45%–55% V.O2max), and the average heart rate is 135–155 beats/min (70%–85% HRmax), with mean blood lactate <4 mmol/L, subjective fatigue level of 12 to 14 (moderate intensity), and mean metabolic equivalent of 5 to 7 METs. However, average intensity does not effectively reflect the physiological characteristics of tennis matches, and athletes have higher intensity indicators between rounds [24]. Tennis biomechanics research mainly focuses on the strength characteristics of tennis players, the kinematic characteristics of different links of the body in the process of hitting the ball, biomechanical differences between different hitting techniques, tennis player injuries, and biomechanical characteristics of equipment [25]. See Figures 4 and 5.

In tennis, the importance of technical movements is unquestionable; a good batting action can not only create the maximum batting speed for the athlete's batting, but also improve batting control and forehand action. In this study, we will mainly analyze the kinematics and dynamics parameters from the athlete's arrival at the hitting position, from the landing of the right foot to the end of the forward swing; in the results section, we have obtained the parameters of the important moments in the preparation phase and the acceleration swing phase; from these parameters, we can deeply analyze the reasons for the structure and swing performance of tennis players of different levels of forehand.

## 5. Conclusion

The tennis forehand is a continuous process; when the frame is in the part of touching the ball, it is necessary to bend the legs moderately so as to fully spin; at this time, the foot is off the ground, but the body is still in the coordinated chain of power and speed transmission. During the whole process of touching the ball, the hips, body, and shoulders form the basic elements of maintaining balance. When the ball is touched, the momentum of the ball and the distance of the ball from the center of the racket produce a rotational torque, making the speed generated by the head of the racket as an angular movement from the bulky part of the body (slower movements, such as the trunk) be transferred to the light part (extremely fast movement, such as the wrist), to maintain the weight *x* speed equation and so on. In addition, the head and shoulders should also coordinate to maintain balance during the touch of the ball. Controlling the entire coordination chain and its components, and being able to accurately determine the ball's flight path, will be beneficial to improve the hitting effect. To sum up, the touch link in the tennis forehand process must make full use of the coordination chain of the human body; that is, the four parts of the legs, hips, upper body, and head and shoulders work in a coordinated and orderly manner to overcome inertia and maintain balance; using the reaction force, the large muscle groups contract and store elastic potential energy, and the small muscle groups are precisely controlled, so that the power of the whole body can be smoothly transmitted to the racket; the perfect combination of linear momentum and angular momentum creates a good shot at the right shot.

## Figures and Tables

**Figure 1:** Human coordination chain diagram. For different shot types, control the angle between the racket and the ground.

**Figure 2:** Distribution of round time in tennis matches. The player needs to do 300–500 high-intensity exercises, and the total running distance of the game is 1100–3600 m.

**Figure 3:** Distribution of interval time in tennis matches. The player needs to do 300–500 high-intensity exercises, and the total running distance of the game is 1100–3600 m.

**Figure 4:** Occurrences of different acceleration intervals for national-level tennis players. Tennis biomechanics research mainly focuses on the strength characteristics of tennis players.

**Figure 5:** Occurrences of different acceleration intervals for tennis players at the regional level. Tennis biomechanics research mainly focuses on the strength characteristics of tennis players.

**Table 1:** Correct actions when touching the ball.

Body parts	Body movement	Biomechanical effect	Action essentials
Legs	Fully extended	Promote the formation of angular momentum	Fully extended
Hip	Keep shoulders in line	Balance at the hips, upper body, and shoulders	Keep balance and turn fully
Upper body	Proper use of body parts; grip the racket tightly to prevent the hit point from straying from the sweet spot and creating a torque master in the reality	Correct use of the human body coordination chain, the racket head drives the ball to generate linear momentum and angular momentum	Grip not stiff; rhythmic and reasonable hitting
Head and shoulders	Keep head and shoulders in a straight line; shoulder drive arm rotation	Head and shoulder coordination for balance	Watch the ball

**Table 2:** Common wrong actions when touching the ball.

Body parts	Wrong action
Legs	Excessive knee flexion at impact
Hip	Hip and shoulder end in a straight line
Upper body	Wrists are loose when touching the ball, arms are farther away from the body
Head and chest	Head down, do not look at the ball

## Data Availability

The data used to support the findings of this study are available from the corresponding author upon request.
